The article "In Vitro Antibacterial Activity of Myrtus communis L. and Marrubium vulgare L. Leaves against Aggregatibacter actinomycetemcomitans and Eikenella corrodens" was published in 2021. Journal: Evid Based Complement Alternat Med.

# In Vitro Antibacterial Activity of *Myrtus communis* L. and *Marrubium vulgare* L. Leaves against *Aggregatibacter actinomycetemcomitans* and *Eikenella corrodens*

**DOI:** 10.1155/2021/8351332

**Published:** 2021-10-19

**Authors:** Kaoutar Dib, Yahia Cherrah, Sana Rida, Abdelkarim Filali-Maltouf, OumKeltoum Ennibi

**Affiliations:** ^1^Laboratory of Microbiology and Molecular Biology, Faculty of Sciences, Mohammed V University in Rabat, Rabat, Morocco; ^2^Laboratory of Pharmacology and Toxicology, Faculty of Medicine and Pharmacy, Mohammed V University in Rabat, Rabat, Morocco; ^3^Research Laboratory on Oral Biology and Biotechnology, Faculty of Dental Medicine, Mohammed V University in Rabat, Rabat, Morocco

## Abstract

**Materials and Methods:**

Clinical strains of *Aggregatibacter actinomycetemcomitans* and *Eikenella corrodens* and two reference strains of *A. actinomycetemcomitans* were tested. The antibacterial activity of each studied plant extract was evaluated using agar diffusion and broth microdilution assays.

**Results:**

Both aqueous and methanolic extracts of *M. communis* exhibited high antibacterial activity against periodontal pathogens as compared to *M. vulgare* extracts. At concentrations of 2.5-0.32 mg/disc, inhibition zones of the methanolic extract of *M. communis* ranged from 19.66 ± 0.57 to 12.33 ± 0.57 mm. The methanolic extract of *M. vulgare* showed at concentrations of 5-0.63 mg/disc inhibition zones ranging from 15.66 ± 0.57 to 12 ± 0.00 mm. Its aqueous extract at concentration of 0.63 mg/disc showed no antimicrobial activity against the clinical and reference strain of *A. actinomycetemcomitans. Conclusion*. This study showed that methanolic and aqueous extracts of *M. communis* and *M. vulgare* have in vitro an antibacterial activity against periodontal pathogens. They could be use as ingredients of an oral antimicrobial agent for prevention or treatment of periodontal diseases. Further research on isolating the compounds from these plant extracts and their toxicity effect could be conducted.

## 1. Introduction

Periodontitis is a chronic inflammatory disease that leads to periodontal attachment loss and alveolar bone destruction, which may gradually lead to tooth loss if left untreated. Periodontitis known as “chronic” and “aggressive” periodontitis is currently grouped in one category named “periodontitis” [1]. Many bacterial species associated with periodontitis have been identified in subgingival plaque samples such as *Aggregatibacter actinomycetemcomitans*, *Porphyromonas gingivalis*, *Prevotella intermedia*, *Tannerella forsythia*, *Fusobacterium nucleatum*, *Campylobacter rectus*, and *Eikenella corrodens* [2, 3]*. A. actinomycetemcomitans* is strongly associated with periodontitis, and its pathogenicity is related to the production of numerous virulence factors [4]. *E. corrodens* has also been implicated in destructive periodontal diseases [5].

The article "In Vitro Antibacterial Activity of Myrtus communis L. and Marrubium vulgare L. Leaves against Aggregatibacter actinomycetemcomitans and Eikenella corrodens" was published in 2021. Journal: Evid Based Complement Alternat Med.

Management of this disease is based on mechanical periodontal debridement either none surgically or surgically. In some situations, adjunctive antibacterial treatments are necessary to control biofilm accumulation. However, because of the increasing bacterial resistance and the side effects of antimicrobial agents commonly used in periodontal treatment [6], natural antimicrobial agents have generated a great interest at the global level. Indeed, medicinal plants and their natural compounds may possess antibacterial, antioxidant, and anti-inflammatory activities, which thereby may have real benefits on oral health [7, 8].

Among the wide variety of medicinal plants used worldwide, *Myrtus communis* L. (Myrtaceae), commonly known as myrtle, and *Marrubium vulgare* L. (Lamiaceae), known as “white horehound,” are wide-spreading in the Mediterranean region [9]. It had been reported that these two plants possess several properties, inter alia, antibacterial, anti-inflammatory, analgesic, antioxidant, and antidiabetic [10–13]. In Morocco, *M. communis* and *M. vulgare* are known as “Rihane” and “Merriwut,” respectively. Infusion and decoction from the leaves of *M. communis* are traditionally used for the treatment of respiratory diseases, diarrhoea [14], heart weakness, and digestive disturbances [15]. The leaves of myrtle have been reported to be used as a mouthwash for the treatment of halitosis [16], while its fruits are chewed for gingivitis and mouth ulcers [14]. A decoction from the leaves of *M. vulgare* is used as antidiabetic and can also be chewed for toothache [14]. Additionally, it had been reported that *M. vulgare* is prescribed by Moroccan traditional healers for halitosis [17].

Many studies reported the antibacterial activity of *M. communis* essential oil and *M. vulgare* essential oil against oral pathogens [18–21]. Nevertheless, insufficient data on the antimicrobial effect of the crude extracts of these plants, on periodontal pathogens, are available. Hence, this study aimed to test the antibacterial activity of *M. communis* and *M. vulgare* leaf extracts against selected periodontal pathogens, namely, *A. actinomycetemcomitans* and *E. corrodens*.

## 2. Materials and Methods

The research was conducted in accordance with the Ethical Principles for Medical Research involving human subjects. The approval was obtained from the Biomedical Research Ethics Committee (CERB) of the Faculty of Medicine and Pharmacy of the Mohammed V University in Rabat (n° 54/2018). A total of 10 subjects aged between 20–50 years were recruited from the department of periodontology at the Center of Dental Consultations and Treatments in Rabat. The inclusion criteria were as follows: patients who had a periodontitis and who accepted to participate to the study and signed informant consent. The exclusion criteria were pregnant and lactating women, smokers, and patients who had received systemic antibiotic or periodontal treatment within the last 6 months.

The article "In Vitro Antibacterial Activity of Myrtus communis L. and Marrubium vulgare L. Leaves against Aggregatibacter actinomycetemcomitans and Eikenella corrodens" was published in 2021. Journal: Evid Based Complement Alternat Med.

In these patients, subgingival plaque samples were taken from the deepest periodontal pockets using sterile paper points. The pooled samples were placed in small vials with 1.5 ml of Phosphate Buffer Saline (PBS) and transferred for processing at the Laboratory of Oral Biology and Biotechnology, Faculty of Dental Medicine, Mohammed V University, Rabat.

### 2.1. Plant Materials

*M. communis* was collected from the river Oued Sra in Taounate (in the Rif Mountains region of northern Morocco) during the fall season (October–December). *M. vulgare* was collected during the same period along the Sebou River in Kenitra (northern Morocco). They were identified at the Scientific Institute in Rabat, and the voucher specimens were deposited at the National Herbarium of the Scientific Institute in Rabat, under No. 110498 and No. 110285 for *M. communis* and *M. vulgare*, respectively.

The plants were washed and shade dried for 2 weeks at room temperature. Then, the dried leaves were milled in a mixer, and the powder was stored in an airtight container until use.

#### 2.1.1. Preparation of Aqueous Extracts

50 g of dry powdered leaves of *M. communis* and *M. vulgare* were mixed with 500 ml of sterile distilled water and boiled for 15 min at 100°C. Each extract was filtered by using Wattman filter paper No. 1, and the filtrate was dried under reduced pressure by using a rotary evaporator at 60°C [22]. Then, the aqueous extracts were lyophilized and stored at −20°C until use.

#### 2.1.2. Preparation of Methanolic Extracts

For *M. communis*, the powder from dry leaves was extracted using Soxhlet extraction with 95% methanol for 6 hours with the ratio of 10 : 1(v/w) of solvent [23]. Dry leaves of *M. vulgare* were extracted by maceration in 95% methanol for 48 hours. Extracts of both plants were then filtered by using Wattman filter paper No. 1 and concentrated under reduced pressure using a rotary evaporator at 40°C [24]. Dried methanolic extracts were stored at −20°C for further use.

### 2.2. Microbial Strains

The antibacterial activity of *M. communis* and *M. vulgare* leaf extracts was tested on the following bacteria: clinical strains of *Aggregatibacter actinomycetemcomitans*, *Eikenella corrodens* and 2 reference strains of *A. actinomycetemcomitans* «ATCC 43718» and Y4 «ATCC43718».

The article "In Vitro Antibacterial Activity of Myrtus communis L. and Marrubium vulgare L. Leaves against Aggregatibacter actinomycetemcomitans and Eikenella corrodens" was published in 2021. Journal: Evid Based Complement Alternat Med.

A selective medium “Dentaid-1” was prepared to isolate *A. actinomycetemcomitans* by using Brain Heart Infusion agar supplemented with 5 g of yeast extract, 1.5 g of sodium fumarate, and 1 g of sodium formate per litre. The medium was autoclaved for 15 min at 121°C. Vancomycin was added to a final concentration of 9 *µ*g/mL [25].

The samples were vortexed for 2 min and seeded into the culture media Dentaid-1 for isolation of *A. actinomycetemcomitans* and blood agar culture media for isolation of *E. corrodens.* The inoculated plates were incubated into an anaerobic environment at 37°C under 5% CO_2_ for 3 to 5 days. Identification of the isolates was performed based on guidelines in the manual of Clinical Microbiology [26], i.e., colony morphology, gram staining, and biochemical tests.

Strains were stored at −80°C in Brain Heart Infusion broth with 20% glycerol at the Laboratory of Oral Biology and Biotechnology, Faculty of Dental Medicine, Mohammed V University, Rabat.

### 2.3. Antibacterial Assays

The antibacterial activity of aqueous and methanolic extracts of *M. communis* and *M. vulgare* was evaluated qualitatively and quantitatively by standard agar disk diffusion and broth microdilution according to the Clinical and Laboratory Standards Institute (CLSI) recommendations [27, 28].

The aqueous and methanolic extracts were dissolved in sterile distilled water and 10% dimethyl sulfoxide (DMSO), to determine the concentration of 100 mg/ml and 200 mg/ml as a stock solution for *M. communis* and *M. vulgare*, respectively.

#### 2.3.1. Agar Disk Diffusion

The antimicrobial activity of plant extracts was evaluated by agar disk diffusion as previously described [23]. The stock solutions were diluted to 12.5–100 mg/ml at a final concentration for *M. communis* and 25–200 mg/ml for *M. vulgare* and used for antimicrobial testing.

Colonies of bacterial strains were picked from overnight pure culture on a nonselective medium and were suspended in 0.85% NaCl. The suspension of each bacterial strain was standardized with a 0.5 Mc Farland density (1 × 10^8^ colony-forming unit (CFU)/ml) using Sensititre^®^Nephelometer. The inoculum of each bacterial suspension was used within 15 min of preparation and was swabbed in three directions over the entire surface of blood agar plates.

Blank filter paper disks (6 mm in diameter, Oxoid) were impregnated with 25 *µ*l of each plant extract at various concentrations and left to dry for 2 hours before applying them over the test plates. Disks impregnated with 25 *µ*l of sterilized distilled water and 10% DMSO were used as negative controls for aqueous and methanolic extracts, respectively, whereas Doxycycline (30 *µ*g/disc, Oxoid) was used as a positive control. Doxycycline, as a reference antibiotic, showed an efficacy either on *A. actinomycetemcomitans* or *E. corrodens* [29, 30] in in vitro studies.

The article "In Vitro Antibacterial Activity of Myrtus communis L. and Marrubium vulgare L. Leaves against Aggregatibacter actinomycetemcomitans and Eikenella corrodens" was published in 2021. Journal: Evid Based Complement Alternat Med.

The plates were incubated at 37°C, 5% CO_2_ for 48 hr, and after incubation, we measured the diameters of the zone of inhibition in millimetres. All experiments were repeated three times at each concentration of extracts.

#### 2.3.2. Broth Microdilution

The Minimum Inhibitory Concentration (MIC) and the Minimum Bactericidal Concentration (MBC) values of extracts were determined by broth microdilution as previously described [31]. From stock solutions of each extract, two-fold serial dilutions were prepared in Brain Heart Infusion broth (BHI) to obtain concentrations ranging from 50 to 0.19 mg/ml for *M. communis* and 100 to 0,39 mg/ml for *M. vulgare*. 50 *µ*l of each dilution was dispensed into the wells 1 to 9 of a 96-well microtitre plate (Figure 1). The inoculum of each microorganism was prepared by direct suspension of overnight colonies into BHI broth. The suspension was adjusted to equal the turbidity of a 0.5 Mc Farland standard using a nephelometer. Then, 50 *µ*l of each microorganism suspension was added to wells 1 to 10 for a final volume of 0.1 ml.

Control wells were included. An inoculated well with broth but not extracts was used as a positive control to check growth control (well 10), whereas uninoculated wells filled with the extracts and BHI broth served as negative controls. Solvent and medium controls were also used. After incubation at 37°C, 5% CO_2_ for 48 hr, we added 20 *µ*l of Triphenyl Tetrazolium Chloride (TTC, Oxoid) 0.1% solution, and we incubated the plate again for 2 hours [32]. Then, the growth in wells was observed to determine the minimal inhibitory concentration which is the lowest concentration of the extract that inhibits the visible growth of the tested bacteria.

The minimal bactericidal concentration was determined by plating an aliquot of each well that had no color change of indicator, onto blood agar plates, and incubated for 48 hr at 37°C under 5% CO_2_. After incubation, the MBC was recorded at the lowest concentration of the extract that could kill 99.9% of each microorganism on the agar plate. The MIC and MBC assays were repeated three times for each extract.

### 2.4. Statistical Analysis

The data were analyzed using the Statistical Package for the Social Sciences (SPSS). The zone of inhibition values of all extracts at different concentrations were expressed as mean ± standard deviation (SD). Descriptive statistics were performed, and data were analyzed using one-way analysis of variance (ANOVA) and Bonferroni post hoc. Differences between means of inhibition zone diameters of the extracts of both plants were considered statistically significant when the *p* value was less than 5% (*p* < 0,05).

The article "In Vitro Antibacterial Activity of Myrtus communis L. and Marrubium vulgare L. Leaves against Aggregatibacter actinomycetemcomitans and Eikenella corrodens" was published in 2021. Journal: Evid Based Complement Alternat Med.

## 3. Results

The methanolic and aqueous extracts of *M. communis* and *M. vulgare* exhibited antibacterial activity against clinical and reference strains of *A. actinomycetemcomitans* and clinical strains of *E. corrodens.* Both *M. communis* and *M. vulgare* extracts showed that the zone of inhibition increased as the concentrations of extracts increased. The aqueous extract of *M. vulgare* at a concentration of 0.63 mg/disc showed no antimicrobial activity against the clinical and reference strain of *A. actinomycetemcomitans.*

Clinical strains and reference strains of *A. actinomycetemcomitans* had the same susceptibility to extracts of both plants, and there was no statistically significant difference (*p* < 0,05). All bacterial strains showed susceptibility to doxycycline. The inhibition zone data of two plant extracts are summarized in Tables 1 and 2 .

The results of the Minimum Inhibitory Concentrations (MICs) determined by microbroth dilution and the Minimum Bactericidal Concentrations (MBCs) obtained from the plates are showed in Table 3. The MICs of the methanolic and aqueous extract of *M. communis* ranged between 0.19–3.12 mg/ml against all periodontal pathogens. The MICs of the methanolic extract of *M. vulgare* ranged between 1.56–3.12 mg/ml, whereas the MICs of its aqueous extract ranged between 25–50 mg/ml.

## 4. Discussion

The present study showed that the aqueous and methanolic extracts of *M. communis* and *M. vulgare* had an antibacterial activity against the tested strains, i.e., *A. actinomycetemcomitans* and *E. corrodens*.

Although aqueous and methanolic extracts of *M. communis* were active against all microorganisms tested in all concentrations, methanolic extract was significantly more effective than aqueous extract. Both extracts exhibited high antibacterial activity as compared to the methanolic and aqueous extract of *M. vulgare*. The methanolic extract of *M. vulgare was* found to be more effective when compared with its aqueous extract. These results may be attributed to a better solubility of the active compounds in organic solvents such as methanol and ethanol. Furthermore, it was shown that the highest extraction of total phenolic compounds from *M. vulgare* leaves was obtained by methanol [33].

An antibacterial agent is considered to have a bactericidal effect if the ratio of MBC/MIC is ≤4 and having a bacteriostatic effect if the ratio is >4 [34, 35]. For the tested plant extracts, the MBC/MIC ratio was less than four except for the aqueous extract of *M. vulgare*. Thus, the aqueous and methanolic extracts of *M. communis* and the methanolic extract of *M. vulgare* showed a bactericidal activity, while the aqueous extract of *M. vulgare* showed a bacteriostatic effect.

The article "In Vitro Antibacterial Activity of Myrtus communis L. and Marrubium vulgare L. Leaves against Aggregatibacter actinomycetemcomitans and Eikenella corrodens" was published in 2021. Journal: Evid Based Complement Alternat Med.

The antimicrobial activity of *M. communis* and *M. vulgare* against periodontal pathogens may be attributed to their active components. Indeed, leaves of *M. communis* are known to contain polyphenolic compounds, tannins, and flavonoid glycosides [36]. A chromatographic HPLC profile of the myrtle leaves identified 15 new phenolic compounds [37]. It had shown that these different compounds possess an antibacterial activity [38–41]. Regarding *M. vulgare*, the principal component is diterpenes labdane marrubium, and it contains also a variety of compounds, e.g., alkaloids, steroids, terpenes, and tannins [12]. The antibacterial activity of these various compounds has been reported in some studies [42–44].

These plant extracts may probably act as an antimicrobial agent that involves specific mechanisms toward bacterial cells. Indeed, they may interfere with cell wall synthesis and protein synthesis and can also affect cytoplasmic membrane and cell metabolism [45].

The antibacterial activity of *M. communis* leaf extracts has been reported against Gram-positive bacteria (*Staphylococcus aureus, Micrococcus luteus, Streptococcus pneumoniae, Streptococcus pyogenes, Streptococcus agalactiae,* and *Listeria monocytogenes*) and Gram-negative bacteria (*Escherichia coli, Proteus vulgaris, Pseudomonas aeruginosa,* and *Campylobacter jejuni*) [46]. It had been also reported that the hydroalcoholic extract of myrtle leaves had the great effect on *Staphylococcus aureus* and *Vibrio chloreae* [47]. Additionally, Rahimvand et al. [48] showed that the aqueous and methanolic extracts of myrtle leaves had an antimicrobial effect against the reference strains of *A. actinomycetemcomitans*, *Porphyromonas gingivalis*, and *Prevotella intermedia*. Other studies reported the antibacterial activity in vitro of polyherbal toothpaste containing leaf extracts of *M. communis* against oral pathogens (*Streptococcus mutans, Lactobacillus casei, S. sanguis, S. salivarius, and Candida albicans*) and the clinical efficacy of a paste containing *M. communis* leaves in the treatment of recurrent aphthous stomatitis [49, 50].

Previous studies have shown an antimicrobial activity of *M. vulgare* extracts against pathogenic microorganisms, e.g., *Escherichia coli*, *Bacillus cereus*, *Proteus mirabilis*, and other bacterial and fungal strains, e.g., *Staphylococcus aureus*, *Klebsiella pneumoniae, Candida albicans*, *Aspergillus flavus*, and *M. tuberculosis* [51–53]. We assume that this study is the first one to assess the antimicrobial efficacy of *M. vulgare* against periodontal pathogens.

The article "In Vitro Antibacterial Activity of Myrtus communis L. and Marrubium vulgare L. Leaves against Aggregatibacter actinomycetemcomitans and Eikenella corrodens" was published in 2021. Journal: Evid Based Complement Alternat Med.

Through this study, we acquire attention to the traditional use of medicinal plants for oral health in Morocco. Indeed, during the last ten years, many studies were particularly interested in the biological activities of medicinal plants on general health, but published national ethnobotanical studies on oral health are limited, and some of them reported that only 2% of medicinal plants are traditionally used for oral hygiene [54, 55]. Compared with the rate of the therapeutic use of plants for other infectious diseases, dental use remains low in most regions of Morocco. For example, in Taounate Province (north of Morocco), only 2.3% of medicinal plants were used traditionally for the mouth and dental hygiene, while 24.9% was used for digestive disorders and 9.8% for the bronchopulmonary system [15]. Diverse plants used in traditional medicine may be interesting for the identification of new antimicrobial agents against relevant periodontal pathogens. Nevertheless, good oral hygiene is a major factor in maintaining periodontal health, and the use of adjuvant agents based on medicinal plants may be a good help for plaque control. Indeed, many herbal drugs and natural products are used as antimicrobial agents in kinds of toothpaste and mouth rinses to reduce plaque accumulation and gingival inflammation [56].

This study showed that *M. communis* and *M. vulgare* possess in vitro antibacterial activity against periodontal pathogens. However, we have only studied the crude extracts of the leaves of these plants, and the active compounds of each plant must be isolated and tested. The bacteria tested were in planktonic culture; thereby, the antimicrobial activity of these plants should be verified against subgingival bacterial biofilm communities. The relationship between different subgingival microorganisms may interfere with their susceptibility to antimicrobial agents. Previous studies have shown that most subgingival bacteria species were resistant to antimicrobials when they are protected by a biofilm structure in comparison with the planktonic bacteria [57, 58].

As periodontitis is a polymicrobial infection, we suggest further analysis of the antibacterial effect of the tested plant extracts against other periodontal pathogens such as bacteria of the red complex or bacteria newly associated with periodontitis and also against periodontal biofilm. The synergistic action of these plant extracts should be considered too. Finally, cells and animal toxicity studies of these plants and their active compounds are to achieve before clinical trials.

The article "In Vitro Antibacterial Activity of Myrtus communis L. and Marrubium vulgare L. Leaves against Aggregatibacter actinomycetemcomitans and Eikenella corrodens" was published in 2021. Journal: Evid Based Complement Alternat Med.

## 5. Conclusions

With the limit of the present study, the extracts of *M. communis* and *M. vulgare* showed an antibacterial effect on *A. actinomycetemcomitans* and *E. corrodens*. This antimicrobial action of natural compounds could serve as a suitable adjunctive agent for the prevention or treatment of periodontal diseases associated with these microorganisms. As periodontitis is associated with a complex multimicrobial biofilm, further analysis is needed for conclusive statement about the potential benefit of the extracts of *M. communis* and *M. vulgare.*

## Figures and Tables

**Figure 1:** Illustration of an example of the 96-well microplate's broth microdilution method for testing the methanolic extract of *M. communis* on a clinical strain of *A. actinomycetemcomitans* (3 test rows A, B, and C) and a clinical strain of *E. corrodens* (3 test rows E, F, and G) for *M. communis* MIC. Wells on column 10 are marked as the positive control (inoculated well with broth but not extracts), and wells on 11 are marked as negative controls (wells filled with the extracts and BHI broth).

**Table 1:** Inhibition zone of aqueous and methanolic extracts of *M. communis* leaves against periodontal pathogens (mm).

Periodontal pathogens	Plant extracts	Concentrations (mg/disc)				*p* value
		2.5	1.25	0.63	0.32	
*A.a* ^1^ clinical strain	MeOH^3^	18 ± 0.00^*∗∗*^	16. ± 1.00	14.33 ± 0.57	12.66 ± 0.57	0.001^*∗*^
	Aqueous	14.66 ± 0.57	13.33 ± 0.57	12.33 ± 0.57	11.33 ± 0.57	0.001^*∗*^

*A.a* ^1^Y4 ATCC 43718	MeOH	19.66 ± 0.57	16.33 ± 0.57	15.33 ± 0.57	13.33 ± 0.57	0.001^*∗*^
	Aqueous	16.33 ± 0.57	14.33 ± 0.57	13.33 ± 0.57	12 ± 1.00	<0.001^*∗*^

*A.a* ^1^ATCC 43718	MeOH	18. ± 0.00	15. ± 0.00	14.33 ± 0.57	12.33 ± 0.57	0.002^*∗*^
	Aqueous	15.66 ± 0.57	13.66 ± 0.57	12.66 ± 0.57	11.66 ± 0.57	<0.001^*∗*^

*E.c* ^2^ clinical strain 1	MeOH	19.33 ± 1.15	15.33 ± 0.57	14 ± 0.00	12.66 ± 0.57	0.003^*∗*^
	Aqueous	14.33 ± 0.57	13 ± 1.00	12.33 ± 0.57	11.66 ± 1.15	0.012^*∗*^

*E.c* ^2^ clinical strain 2	MeOH	18.33 ± 0.57	15.33 ± 0.57	14 ± 1.00	13 ± 0.00	0.002^*∗*^
	Aqueous	14 ± 0.00	13 ± 0.00	12.66 ± 1.15	11.33 ± 0.57	<0.001^*∗*^

*E.c* ^2^ clinical strain 3	MeOH	17.33 ± 0.57	15.00 ± 0.00	14 ± 0.00	12.66 ± 0.57	0.002^*∗*^
	Aqueous	14.33 ± 0.57	13.66 ± 1.15	12 ± 0.00	11.33 ± 0.57	0.012^*∗*^

^*∗*^Test applied- one-way analysis of variance (ANOVA), *p* < 0.05 (statistically significant). ^*∗∗*^All values of inhibition zone are presented as mean ± SD (mm) from three experiments. ^1^*A. actinomycetemcomitans*; ^2^*E. corrodens*; ^3^*methanolic*.

The article "In Vitro Antibacterial Activity of Myrtus communis L. and Marrubium vulgare L. Leaves against Aggregatibacter actinomycetemcomitans and Eikenella corrodens" was published in 2021. Journal: Evid Based Complement Alternat Med.

**Table 2:** Inhibition zone of aqueous and methanolic extracts of *M. vulgare* leaves against periodontal pathogens (mm).

Periodontal pathogens	Plant extracts	Concentrations (mg/disc)				*p* value
		5	2.5	1.25	0.63	
*A.a* ^1^ clinical strain	MeOH^3^	14.66 ± 0.57	14 ± 1.00	13.33 ± 0.57	12.33 ± 0.57	0,010^*∗*^
	Aqueous	13 ± 0.00^*∗∗*^	11.33 ± 0.57	9.33 ± 0.57	NI^4^	0,023^*∗*^

*A.a* ^1^Y4 ATCC 43718	MeOH	15.66 ± 0.57	14 ± 0.00	13.33 ± 0.57	12.33 ± 0.57	<0,001^*∗*^
	Aqueous	13 ± 0.00	11.33 ± 0.57	9.33 ± 0.57	NI^4^	0,023^*∗*^

*A.a* ^1^ATCC 43718	MeOH	15. ± 0.00	13.66 ± 0.57	13 ± 0.00	12. ± 0.00	<0,001^*∗*^
	Aqueous	13.66 ± 0.17	12.66 ± 0.57	11.66 ± 0.57	10.33 ± 0.57	0,002^*∗*^

*E.c* ^2^ clinical strain 1	MeOH	15 ± 0.00	14 ± 0.00	12.66 ± 0.57	12 ± 1.00	0,003^*∗*^
	Aqueous	13.66 ± 0.57	12. ± 0.00	11.33 ± 0.57	10 ± 0.00	<0,001^*∗*^

*E.c* ^2^ clinical strain 2	MeOH	15 ± 0.00	14 ± 1.00	13 ± 0.00	12.33 ± 1.15	0,011^*∗*^
	Aqueous	13.33 ± 0.57	12.33 ± 0.57	12 ± 0.00	10.66 ± 0.57	0,014^*∗*^

*E.c* ^2^ clinical strain 3	MeOH	14.66 ± 0.57	13.66 ± 0.57	12.66 ± 0.57	12 ± 0.00	0,002^*∗*^
	Aqueous	13.33 ± 0.57	12.66 ± 0.57	11.66 ± 0.57	10.33 ± 0.57	0,004^*∗*^

^*∗*^Test applied- one-way analysis of variance (ANOVA), *p* < 0,05 (statistically significant). ^*∗∗*^All values of inhibition zone are presented as mean ± SD (mm) from three experiments. ^1^*A. actinomycetemcomitans*; ^2^*E. corrodens;*^3^*methanolic*; ^4^no inhibition zone.

**Table 3:** Minimum Inhibitory Concentration (MIC) and Minimum Bactericidal Concentration (MBC) of *M. communis* and *M. vulgare* extracts against periodontal pathogens.

Periodontal pathogens	*M. communis*				*M. vulgare*			
	Methanolic		Aqueous		Methanolic		Aqueous	
	MIC^3^ (mg/ml)	MBC^4^ (mg/ml)	MIC (mg/ml)	MBC (mg/ml)	MIC (mg/ml)	MBC (mg/ml)	MIC (mg/ml)	MBC (mg/ml)
*A.a* ^1^ clinical strain	≤0.19	0.39	1.56	3.12	3.12	6.25	50	>100
*A.a* ^1^Y4 ATCC 43718	≤0.19	0.39	0.78	0.78	I.56	3.12	50	100
*A.a* ^1^ATCC 43718	≤0.19	0.39	0.78	1.56	3.12	6.25	25	>100
*E.c* ^2^ clinical strain 1	≤0.19	0,19	3.12	6.25	3.12	3.12	25	100
*E.c* ^2^ clinical strain 2	≤0.19	0.19	3.12	6.25	3.12	6.25	25	100
*E.c* ^2^ clinical strain 3	0,39	0.39	3.12	6.25	3.12	6.25	25	100

^1^ *A. actinomycetemcomitans*; ^2^*E. corrodens*; ^3^minimum inhibitory concentration (mg/ml); ^4^ minimum bactericidal concentration (mg/ml).

## Data Availability

Data supporting the results of our study are included in the manuscript.

## References

[1] Papapanou P. N., Sanz M., Buduneli N. (2018). Periodontitis: consensus report of workgroup 2 of the 2017 world workshop on the classification of periodontal and peri-implant diseases and conditions. *Journal of Periodontology*.

The article "In Vitro Antibacterial Activity of Myrtus communis L. and Marrubium vulgare L. Leaves against Aggregatibacter actinomycetemcomitans and Eikenella corrodens" was published in 2021. Journal: Evid Based Complement Alternat Med.

[2] Jervoe-Storm P.-M., Koltzscher M., Falk W., Dörfler A., Jepsen S. (2005). Comparison of culture and real-time PCR for detection and quantification of five putative periodontopathogenic bacteria in subgingival plaque samples. *Journal of Clinical Periodontology*.

[3] Loomer P. M. (2004). Microbial diagnostic testing in the treatment of periodontal diseases. *Periodontology 2000*.

[4] Raja M., Ummer F., Dhivakar C. P. (2014). *Aggregatibacter actinomycetemcomitans*–a tooth killer?. *Journal of Clinical and Diagnostic Research*.

[5] Haffajee A. D., Socransky S. S. (1994). Microbial etiological agents of destructive periodontal diseases. *Periodontology 2000*.

[6] Serrano C., Torres N., Valdivieso C., Castaño C., Barrera M., Cabrales A. (2009). Antibiotic resistance of periodontal pathogens obtained from frequent antibiotic users. *Acta Odontologica Latinoamericana: AOL*.

[7] M. Varoni E., Lodi G., Sardella A., Carrassi A., Iriti M. (2012). Plant polyphenols and oral health: old phytochemicals for new fields. *Current Medicinal Chemistry*.

[8] Petti S., Scully C. (2009). Polyphenols, oral health and disease: a review. *Journal of Dentistry*.

[9] Sisay M., Gashaw T. (2017). Ethnobotanical, ethnopharmacological, and phytochemical studies of *Myrtus communis linn*: a popular herb in uUnani system of medicine. *Journal of Evidence-Based Complementary & Alternative Medicine*.

[10] Tuberoso C. I. G., Rosa A., Bifulco E. (2010). Chemical composition and antioxidant activities of *Myrtus communis L.* berries extracts. *Food Chemistry*.

[11] Hosseinzadeh H., Khoshdel M., Ghorbani M. (2011). Antinociceptive, anti-inflammatory effects and acute toxicity of aqueous and ethanolic extracts of *Myrtus communis L.* Aerial parts in mice. *Journal of Acupuncture and Meridian Studies*.

[12] Meyre-Silva C., Cechinel-Filho V. (2010). A review of the chemical and pharmacological aspects of the genus *Marrubium*. *Current Pharmaceutical Design*.

[13] Amri B., Martino E., Vitulo F. (2017). *Marrubium vulgare L.* leave extract: phytochemical composition, antioxidant and wound healing properties. *Molecules*.

[14] Bellakhdar J. (1997). *La Pharmacopée Marocaine Traditionnelle. Médecine Arab ancienne savoirs Populaires*.

[15] El-Hilaly J., Hmammouchi M., Lyoussi B. (2003). Ethnobotanical studies and economic evaluation of medicinal plants in Taounate province (Northern Morocco). *Journal of Ethnopharmacology*.

[16] Tahri N., EL Basti A., Zidane L., Rochdi A., Douira A. (2012). Etude ethnobotanique Des plantes médicinales Dans La province de Settat (Maroc). *Kastamonu University Journal of Forestry Faculty*.

The article "In Vitro Antibacterial Activity of Myrtus communis L. and Marrubium vulgare L. Leaves against Aggregatibacter actinomycetemcomitans and Eikenella corrodens" was published in 2021. Journal: Evid Based Complement Alternat Med.

[17] Akkaoui S., Ennibi O. K. (2017). Use of traditional plants in management of halitosis in a Moroccan population. *Journal of intercultural ethnopharmacology*.

[18] Hedayati A., Khosropanah H., Bazargani A., Abed M., Emami A. (2013). Assessing the antimicrobial effect of the essential Oil of *Myrtus communis* on the clinical isolates of *Porphyromonas gingivalis*: an in vitro study. *Jundishapur Journal of Natural Pharmaceutical Products*.

[19] Fani M. M., Kohanteb J., Araghizadeh A. (2014). Inhibitory activity of Myrtus communis oil on some clinically isolated oral pathogens. *Medical Principles and Practice*.

[20] Laouer H., Yabrir B., Djeridane A., Yousfi M., Beldovini N., Lamamra M. (2009). Composition, antioxidant and antimicrobial activities of the essential oil of *Marrubium deserti*. *Natural product communications*.

[21] Zarai Z., Kadri A., Ben Chobba I. (2011). The in-vitro evaluation of antibacterial, antifungal and cytotoxic properties of *Marrubium vulgare L.* essential oil grown in Tunisia. *Lipids in Health and Disease*.

[22] Kandil O., Radwan N. M., Hassan A. B., Amer A. M. M., El-Banna H. A., Amer W. M. M. (1994). Extracts and fractions of *Thymus capitatus* exhibit antimicrobial activities. *Journal of Ethnopharmacology*.

[23] Salie F., Eagles P. F. K., Leng H. M. J. (1996). Preliminary antimicrobial screening of four South African *Asteraceae* species. *Journal of Ethnopharmacology*.

[24] Nostro A., Germano M. P., D’Angelo V., Marino A., Cannatelli M. A. (2000). Extraction methods and bioautography for evaluation of medicinal plant antimicrobial activity. *Letters in Applied Microbiology*.

[25] Alsina M., Olle E., Frias J. (2001). Improved, low-cost selective culture medium for *Actinobacillus actinomycetemcomitans*. *Journal of Clinical Microbiology*.

[26] Zbinden R. (2015). Aggregatibacter, capnocytophaga, Eikenella, kingella, pasteurella, and other fastidious or rarely encountered gram-negative rods. *Manual of Clinical Microbiology*.

[27] CLSI (2012). *Performance Standards for Antimicrobial Disk Susceptibility Tests; Approved Standard-Eleventh Edition*.

[28] CLSI (2012). *Methods for Antimicrobial Susceptibility Testing of Anaerobic Bacteria; Approved Standard- Eighth Edition*.

[29] Müller H.-P., Holderrieth S., Burkhardt U., Höffler U. (2002). In vitro antimicrobial susceptibility of oral strains of Actinobacillus actinomycetemcomitans to seven antibiotics. *Journal of Clinical Periodontology*.

[30] Tsaousoglou P., Nietzsche S., Cachovan G., Sculean A., Eick S. (2014). Antibacterial activity of moxifloxacin on bacteria associated with periodontitis within a biofilm. *Journal of Medical Microbiology*.

The article "In Vitro Antibacterial Activity of Myrtus communis L. and Marrubium vulgare L. Leaves against Aggregatibacter actinomycetemcomitans and Eikenella corrodens" was published in 2021. Journal: Evid Based Complement Alternat Med.

[31] Basri D. F., Tan L. S., Shafiei Z., Zin N. M (2012). Vitro antibacterial activity of galls of *Quercus infectoria olivier* against oral pathogens. *Evidence-Based Complementary and Alternative Medicine*.

[32] Eloff J. N. (1998). A sensitive and quick microplate method to determine the minimal inhibitory concentration of plant extracts for bacteria. *Planta Medica*.

[33] Bouterfas K., Mehdadi Z., Benmansour D., Khaled M. B., Bouterfas M., Latreche A. (2014). Optimization of extraction conditions of some phenolic compounds from white horehound (*Marrubium vulgare L.*) leaves. *International Journal of Organic Chemistry*.

[34] Abedon S. (2011). Phage therapy pharmacology. *Advances in Applied Microbiology*.

[35] Levison M. E., Levison J. H. (2009). Pharmacokinetics and pharmacodynamics of antibacterial agents. *Infectious Disease Clinics of North America*.

[36] Yoshimura M., Amakura Y., Tokuhara M., Yoshida T. (2008). Polyphenolic compounds isolated from the leaves of *Myrtus communis*. *Journal of Natural Medicines*.

[37] Díaz-de-Cerio E., Arráez-Román D., Segura-Carretero A. (2018). Establishment of pressurized-liquid extraction by response surface methodology approach coupled to HPLC-DAD-TOF-MS for the determination of phenolic compounds of myrtle leaves. *Analytical and Bioanalytical Chemistry*.

[38] Appendino G., Maxia L., Bettoni P. (2006). Antibacterial galloylated alkylphloroglucinol glucosides from myrtle (*Myrtus communis*). *Journal of Natural Products*.

[39] Nassar M., Aboutabl E.-S., Ahmed R., El-Khrisy E.-D., Ibrahim K., Sleem A. (2010). Secondary metabolites and bioactivities ofMyrtus communis. *Pharmacognosy Research*.

[40] Aleksic V., Knezevic P. (2014). Antimicrobial and antioxidative activity of extracts and essential oils of *Myrtus communis L*. *Microbiological Research*.

[41] Cottiglia F., Casu L., Leonti M. (2012). Cytotoxic phloroglucinols from the leaves of *Myrtus communis*. *Journal of Natural Products*.

[42] Kurbatova N. V., Muzychkina R. A., Mukhitdinov N., Parshina G. N. (2003). Comparative phytochemical investigation of the composition and content of biologically active substances in *Marrubium vulgare* and *M. alternidens*. *Chemistry of Natural Compounds*.

[43] Djahra A. B., Bordjiba O., Benkherara S. (2013). Extraction, séparation et activité antibactérienne des tanins de marrube blanc (*Marrubium vulgare L*). *Phytothérapie*.

[44] Masoodi M., Ali Z., Liang S., Yin H., Wang W., Khan I. A. (2015). Labdane diterpenoids from *Marrubium vulgare*. *Phytochemistry Letters*.

[45] Sandle T. (2016). Antibiotics and preservatives. *Pharmaceutical Microbiology: Essentials for Quality Assurance and Quality Control*.

The article "In Vitro Antibacterial Activity of Myrtus communis L. and Marrubium vulgare L. Leaves against Aggregatibacter actinomycetemcomitans and Eikenella corrodens" was published in 2021. Journal: Evid Based Complement Alternat Med.

[46] Mansouri S., Foroumadi A., Ghaneie T., Najar A. G. (2001). Antibacterial activity of the crude extracts and fractionated constituents of *Myrtus communis*. *Pharmaceutical Biology*.

[47] Taheri A., Seyfan A., Jalalinezhad S., Nasery F. (2013). Antibacterial effect of *Myrtus communis* hydro-alcoholic extract on pathogenic bacteria. *Zahedan Journal of Research in Medical Sciences*.

[48] Rahimvand L., Niakan M., Naderi N. J. (2018). The antibacterial effect of aquatic and methanolic extract of *Myrtus communis* on *Actinobacillus actinomycetemcomitans, Porphyromonas gingivalis* and *Prevotella intermedia*. *Iranian Journal of Microbiology*.

[49] Sadeghi-Nejad B., Moghimipour E., Naanaie S. Y., Nezarat S. (2018). Antifungal and antibacterial activities of polyherbal toothpaste against oral pathogens, in vitro. *Current Medical Mycology*.

[50] Babaee N., Mansourian A., Momen-Heravi F., Moghadamnia A., Momen-Beitollahi J. (2010). The efficacy of a paste containing *Myrtus communis* (Myrtle) in the management of recurrent aphthous stomatitis: a randomized controlled trial. *Clinical Oral Investigations*.

[51] Bouterfas K., Mehdadi Z., Elaoufi M. M., Aouad L., Latreche A., Benchiha W. (2018). In vitro antibacterial activity of flavonoids extracts from three Algerian horehound (*Marrubium vulgare L.*) leaves. *Oriental Pharmacy and Experimental Medicine*.

[52] Al-Tohamy R., Ali S. S., Saad-Allah K. (2018). Phytochemical analysis and assessment of antioxidant and antimicrobial activities of some medicinal plant species from Egyptian flora. *Journal of Applied Biomedicine*.

[53] Molina-Salinas G. M., Ramos-Guerra M. C., Vargas-Villarreal J., Mata-Cárdenas B. D., Becerril-Montes P., Said-Fernández S. (2006). Bactericidal activity of organic extracts from *Flourensia cernua DC* against strains of *Mycobacterium tuberculosis*. *Archives of Medical Research*.

[54] Hachi M., Hachi T., Belahbib N., Dahmani J., Zidane L. (2015). Contrbution à l’étude floristique et ethnobotanique de la flore médicinale utilisée au niveau de la ville de Khenifra (Maroc). *International Journal of Innovation and Applied Studies*.

[55] El Hafian M., Benlandini N., Elyacoubi H., Zidane L., Rochdi A. (2014). Étude floristique et ethnobotanique des plantes médicinales utilisées au niveau de la préfecture d’Agadir-Ida-Outanane (Maroc). *Journal of Applied Biosciences*.

[56] Groppo F. C., Bergamaschi C. D. C., Cogo K., Franz-Montan M., Motta R. H. L., Andrade E. D. D. (2008). Use of phytotherapy in dentistry. *Phytotherapy Research*.

[57] Kolenbrander P. E., Palmer R. J., Rickard A. H., Jakubovics N. S., Chalmers N. I., Diaz P. I. (2006). Bacterial interactions and successions during plaque development. *Periodontology 2000*.

The article "In Vitro Antibacterial Activity of Myrtus communis L. and Marrubium vulgare L. Leaves against Aggregatibacter actinomycetemcomitans and Eikenella corrodens" was published in 2021. Journal: Evid Based Complement Alternat Med.

[58] Sedlacek M. J., Walker C. (2007). Antibiotic resistance in an in vitro subgingival biofilm model. *Oral Microbiology and Immunology*.

